# Research on Multi-Time-Delay Gene Regulation Network Based on Fuzzy Label Propagation

**DOI:** 10.1155/2020/2389527

**Published:** 2020-03-11

**Authors:** Haigang Li, Qian Zhang, Ming Li

**Affiliations:** School of Information and Control Engineering, China University of Mining and Technology, Xuzhou, Jiangsu 221116, China

## Abstract

In view of time delay existing in gene regulation, by using the analysis idea and methods of complex network, this paper proposes a multi-time-delay gene regulation network analysis method based on the fuzzy label propagation. The algorithm takes the relative change trend coefficient, the correlation coefficient, and the mutual information as the similarity measurement indexes for the gene pair, fully reflecting the correlation of gene pairs and simultaneously obtaining the gene regulation relationship and the time delay through the fuzzy label propagation algorithm of the semisupervised learning. Experimental results of the cell cycle-regulated genes of yeast show that the proposed construction method of GRN can not only correctly select potential regulation genes but also provide details about the gene regulator model, thereby more accurately constructing gene regulation network.

## 1. Introduction

The interaction between the implicit genes in gene expression data can be used to construct gene regulatory network by analysing gene expression data [1]. The research of gene regulatory network is one of the topics of postgenomic informatics. It mainly analyses gene expression data, uses bioinformatics methods and technologies to identify the topological structure of gene network to deeply understand the structure and function of biology and the mechanism of pathological changes, and understands life phenomena in a systematic framework [2, 3]. Gene network research can be used to reveal the development process and mechanism of biological tissue system and help understand the regulation of internal substances, which can promote people to effectively identify the cause of disease. In particular, the study of human tumor gene regulatory network can make us have a deep understanding of the regulatory relationship of tumor related genes and then provide basis and guidance for tumor gene therapy. Gene regulatory network, as the molecular basis of basic cell life activities, has the biological characteristics of randomness, complexity, spatiotemporal specificity, and dynamic. This makes the construction of gene regulatory network very difficult.

The time-series gene expression data have been widely applied in the research on the gene regulation network, and attention to the time delay has been paid increasingly as the important factor for the gene regulation network construction [4]. The time-delay processing can be generally classified into two types: first type—firstly calculate the time delay among genes, then translate the time-series gene expression data to the calculated time delay to achieve the effect of removing delay, and finally construct the gene regulation network to analyse the regulation relationship among the genes; second type—directly construct the time-delay gene regulation network model and obtain the time delay and the regulation relationship through the time-delay regulation network method [5]. In the first type of analysis, Ahsen et al. [6] obtained the phase and frequency of two gene expression data in the frequency domain through the frequency domain change and calculated the time delay on the basis of the relationship between the phase and the frequency. Huang et al. [7] obtained the mutual time delay among 101 genes by using this time-delay estimation method, constructed the gene regulation network by adopting the concept of community detection, and obtained the better result. The delay time obtained by this method is not always the integer multiple of time interval, and it is necessary to obtain the delay removed gene expression value by using the curve fitting method, which is not conducive to the follow-up study.

The regulation time of gene expression in cells is not synchronous, and the regulation delay length is also different [8]. The existing dynamic Bayesian network model of gene expression regulation network based on time-series gene expression data is difficult to model the asynchronous multi-time-delay regulation relationship [9]. In order to solve this urgent problem, this paper proposes a semisupervised learning method that can accurately model the asynchronous and multi-time-delay regulatory relationship between genes. It can learn the gene expression regulatory network with asynchronous and multi-time-delay characteristics from the time-series expression data of gene chip. In the learning process, it can use the known class data and the unknown class data to obtain more information and have better learning effect.

## 2. Related Work

The reconstruction of gene regulatory network based on expression data is also called reverse engineering or network inference. In recent years, various algorithms have been proposed by analysing gene expression data, such as GA [10], gene programming [11], evolutionary strategies [12], and ACO [13]. However, the GRNs modeled by the above algorithm consist of only a limited number of genes. How to reconstruct large-scale gene regulatory network is still an unknown biological problem.

At present, there are various models to model gene regulatory network. The simplest model is based on Boolean networks. In reverse engineering, Boolean networks are used to infer the underlying topology and the Boolean functions at the nodes from the observed gene expression data. In addition, continuous network is an extension of Boolean network [14], which is also widely used to model gene regulatory network. Nodes still represent the regulatory effect of genes and their connections on gene expression. Genes in biological systems show continuous range of activity levels, and it has been considered that continuous networks can capture some properties of gene regulatory networks that do not exist in Boolean models. Many methods based on continuous networks have been proposed to infer gene regulatory networks, for example, based on linear regression and based on mutual information. In Arachne algorithm, the specific information of each gene pair can be calculated in an appropriate way to get the actual value of mutual information, and compared with the fixed threshold value, a regulatory interaction can be inferred. In addition, many probabilistic graphical models have been proposed to measure the high-order dependence between different gene expression patterns. Bayesian network is one of the most popular methods to infer gene regulatory network. In Bayesian networks, directed acyclic graphs are used to indicate the conditional dependence between random variables [15].

Many researchers think that the time delay among the genes is constant value, and the time delay varies from gene pairs so that the analysis on the multi-time-delay gene regulation network was proposed in succession. To be favorable to construct the gene regulation network, the time delay is normally regarded as the integral multiple of time interval. Based on this, Yang et al. [16] firstly established the time-delay gene expression matrix to dig the time-delay regulation relationship among the genes through the decision tree classifier. Yang [17] constructed the multi-time-delay gene regulation network by using the high-order Markov dynamic Bayesian network. Raja Chowdhury and Chetty [18] constructed the multi-time-delay gene regulation network by using the correlation coefficient method. In this method, the time-delay correlation coefficient among the genes was firstly established, the maximum value of correlation coefficient in each gene pair and the time delay corresponding to this value were obtained through the dynamic threshold method, and finally the maximum value of correlation coefficient in the gene pair was compared with the given threshold to screen the correlation coefficient greater than the threshold and obtain the genes corresponding to these correlation coefficients and the time delay to complete the analysis on the multi-time-delay gene regulation network. This method is simple and can effectively handle the time-delay problem. Aderhold et al. [19] established the time-delay mutual information among the genes and constructed the multi-time-delay gene regulation network through the dynamic Bayesian network: firstly construct the multi-time-delay mutual information matrix to select the larger gene in the mutual information and then complete the analysis on the gene regulation relationship by the dynamic Bayesian network. Better effect has been obtained by this method. However, most of these time-delay methods start from the relationship between genes but ignore the characteristics of genes.

The single metrical scale was used when the similarity among the genes was measured by the above methods. When constructing the gene regulation network, Liu et al. [20] pointed that the single similarity evaluation scale cannot reflect the correlation among the genes very well, so they evaluated the correlation among the genes by using the combined method of correlation coefficient and interquartile range and obtained better gene regulation relationship through the vector analysis by taking the interquartile range of the gene pair as the horizontal ordinate and the correlation coefficient as the vertical coordinate. By reference to [21, 22], this paper combines the multi-time-delay correlation coefficient, the mutual information, and the relative change trend coefficient to construct the new gene pair correlation evaluation matrix and complete the analysis on the multi-time-delay gene regulation network through the semisupervised learning method of fuzzy label propagation.

## 3. Relevant Notes

The time-series gene expression data are denoted as *V*=(*x*_*ij*_)_*N*×*P*_, wherein *x*_*ij*_ expresses the expression value of gene *i* at the time point *j* and *j*=1,2,3,…, *P*. The maximum delay time among the genes is denoted as *A* times the time interval.

### 3.1. Time-Delay Relative Change Trend Coefficient

The matrix obtained by gene expression data discretization is denoted as *D*=(*b*_*ij*_)_*N*×(*P* − 1)_.

(1) $$\begin{array}{c} b_{ij}=\left\{\begin{array}{cc} 1, & \text{if}x_{ij}<x_{i\left(j+1\right)},\\ 0, & \text{if}x_{ij}=x_{i\left(j+1\right)},\\ -1, & \text{if}x_{ij}>x_{i\left(j+1\right)}, \end{array}\right. \end{array}$$

where *j*=1,2,3,…, *P* − 1.

For any two genes *m* and *n* in the dataset, the relative change trend coefficient for the gene *n* and the gene *m* at the time point *j* is denoted as *s*_*mn*,*j*_ after the gene *n* is delayed by *a* unit of time and can be calculated by the following the formulas:

(2) $$\begin{array}{c} b_{mn,j}^{\prime }=b_{mj}\times b_{n\left(j+a\right)},\;j=1,2,3,\ldots ,P-1-a, \end{array}$$

(3) $$\begin{array}{c} s_{mn,j}=b_{mn,j}^{\prime }\times b_{mn,\left(j+1\right)}^{\prime },\;j=1,2,3,\ldots ,P-2-a. \end{array}$$

The value of *s*_*mn*,*j*_ is −1,0,1, wherein 1 indicates the similar change trend of two genes.

The relative change trend of two genes after delay is graded. The number of values equal to 1 is denoted as *s*_*mn*_′, and the relative change trend score for the gene *n* and the gene *m* is denoted as score_*mn*_^*a*^ after the gene *n* is delayed by *a* unit of time.

(4) $$\begin{array}{c} {\text{score}}_{mn}^{a}=\frac{s_{mn}^{\prime }}{P-2-a}. \end{array}$$

### 3.2. Time-Delay Correlation Coefficient

The correlation coefficient for the gene *n* and the gene *m* is denoted as *r*_*mn*_^*a*^ after the gene *n* is delayed by *a* unit of time.

(5) $$\begin{array}{c} r_{mn}^{a}=\frac{\sum_{j=1}^{P-a}\left(x_{mj}-{\bar{x}}_{m}\right)\left(x_{n\left(j+a\right)}-{\bar{x}}_{n}\right)}{\sqrt{\sum_{j=1}^{P-a}{\left(x_{mj}-{\bar{x}}_{m}\right)}^{2}}\sqrt{\sum_{j=1}^{P-a}{\left(x_{n\left(j+a\right)}-{\bar{x}}_{n}\right)}^{2}}}, \end{array}$$

where ${\bar{x}}_{m}$ expresses the mean value of the former *P* − *a* expression values for the gene *m* and ${\bar{x}}_{n}$ expresses the mean value of the latter *P* − *a* expression values for the gene *n*.

### 3.3. Time-Delay Mutual Information

Mutual information expresses the shared information amount between two genes, firstly performing interval partition for the gene expression dataset and then calculating the delay mutual information matrix among the genes. The mutual information for the gene *n* and the gene *m* is denoted as *M*_*mn*_^*a*^ after the gene *n* is delayed by *a* unit of time.

(6) $$\begin{array}{c} M_{mn}^{a}=H\left(m\right)+H\left(n\right)-H\left(m,n\right), \end{array}$$

where *H* is information entropy. The calculation method is as shown in formulas (7) to (9):

(7) $$\begin{array}{c} H\left(m\right)=-\sum p_{m}\log_{2}\left(p_{m}\right), \end{array}$$

(8) $$\begin{array}{c} H\left(n\right)=-\sum p_{n}\log_{2}\left(p_{n}\right), \end{array}$$

(9) $$\begin{array}{c} H\left(m,n\right)=-\sum p_{m,n}\log_{2}\left(p_{m,n}\right), \end{array}$$

where *m* takes the former *P* − *a* expression value and *n* takes the latter *P* − *a* expression value.

### 3.4. Gene Pair Similarity Evaluation Matrix

The gene pair similarity evaluation matrix is *I*=(*i*_*mnfa*_′)_*N*×*N*×3×*A*_, *i*_*mnfa*_′ expresses the expression value of the attribute *f* for the gene *n* and the gene *m* after the gene *n* is delayed by *a* unit of time, and *a*=0,1,…, *A*, wherein the attributes of gene pair are, respectively, relative change trend, correlation coefficient, and mutual information. For the convenience of subsequent analysis, the time-delay similarity evaluation matrix is denoted as *I*=(*i*_*mna*_′)_*N*×*N*×*A*_, wherein *i*_*mna*_′ expresses the similarity sample for the gene *n* and the gene *m* after the gene *n* is delayed by *a* unit of time.

## 4. Multi-Time-Delay Gene Regulation Network Based on Fuzzy Label Propagation

### 4.1. Algorithm Description

The converted datasets are classified by using the fuzzy label propagation algorithm of semisupervised learning. There are two label values: 1 and −1, wherein 1 indicates that the regulation relationship exists between two genes in the gene pair and −1 indicates that there is no regulation relationship.

In the fuzzy label propagation algorithm, firstly divide *I* into the labeled data set *I*_*L*_ and the unlabeled dataset *I*_*U*_ and calculate the similarity *S*_(*mna*)(*m*′*n*′*a*′)_ of any two samples *i*_*mna*_′ and *i*_*m*′*n*′*a*′_′ by using RBP kernel function.

(10) $$\begin{array}{c} S_{\left(mna\right)\left(m^{\prime }n^{\prime }a^{\prime }\right)}=\left\{\begin{array}{cc} 0, & m=m^{\prime },n=n^{\prime },a=a^{\prime },\\ \exp\left(\frac{{\left\|i_{mna}^{\prime }-i_{m^{\prime }n^{\prime }a^{\prime }}^{\prime }\right\|}^{2}}{2\sigma^{2}}\right), & \text{other,} \end{array}\right. \end{array}$$

where *σ* expresses the variance of difference value between two samples.

Express the category of sample *i*_*mna*_′ with the vector *F*_(*mna*)_ of 1 × 2 dimensions:

1. If the sample *i*_*mna*_′ ∈ *I*_*L*_,

(11) $$\begin{array}{c} F_{\left(mna\right)j^{\prime }}=\left\{\begin{array}{cc} 1, & i_{mna}^{\prime }\in \text{the category }j^{\prime },\\ 0, & i_{mna}^{\prime }\notin \text{the category }j^{\prime }, \end{array}\right. \end{array}$$

  where *j*′=1,2.
(2) If the sample *i*_*mna*_′ ∈ *I*_*U*_, the label value of *i*_*mna*_′ is propagated from the *k*′ adjacent samples and the membership that *i*_*mna*_′ belongs to the category *j*′ meets

(12) $$\begin{array}{c} \sum_{i_{m^{\prime }n^{\prime }a^{\prime }}^{\prime }\in N\left(i_{mna}^{\prime }\right)}S_{\left(m^{\prime }n^{\prime }a^{\prime }\right)\left(mna\right)}\left(F_{m^{\prime }n^{\prime }a^{\prime }}-F_{mna}\right)=0, \end{array}$$

where *N*(*i*_*mna*_′) expresses the set composed of *k*′ adjacent samples of *i*_*mna*_′, and the results are obtained from formula (12):

(13) $$\begin{array}{c} F_{mna}=\sum_{i_{m^{\prime }n^{\prime }a^{\prime }}^{\prime }\in N\left(i_{mna}^{\prime }\right)}\frac{S_{\left(m^{\prime }n^{\prime }a^{\prime }\right)\left(mna\right)}}{\sum_{i_{m^{\prime }n^{\prime }a^{\prime }}^{\prime }\in N\left(i_{mna}^{\prime }\right)}S_{\left(m^{\prime }n^{\prime }a^{\prime }\right)\left(mna\right)}}F_{m^{\prime }n^{\prime }a^{\prime }}. \end{array}$$

As the category labels of unknown samples are continuously renewed, *F*_*mna*_ in formula (13) is required to be repeatedly calculated until the fuzzy category label values of all samples are not changed.

Obtain the fuzzy label value *F*=(*F*_*mna*_)_*N*×*N*×*A*_ of all samples and convert the label value matrix by the following formula:

(14) $$\begin{array}{c} F_{mna}=\left\{\begin{array}{cc} F_{mna}, & \text{if}F_{mna}>0,\\ 0, & \text{if}F_{mna}>0. \end{array}\right. \end{array}$$

Convert the label value matrix by the following formula:

(15) $$\begin{array}{c} F_{mna}=\left\{\begin{array}{cc} 1, & \text{if}F_{mna}\neq 0,F_{mna}=\max\left(F_{mn1},F_{mn2},\ldots ,F_{mna}\right),\\ 0, & \text{otherwise.} \end{array}\right. \end{array}$$

The regulation relationship exists between two genes corresponding to the samples with the label value of 1, and the time delay is *a* times the time interval.

### 4.2. Algorithm Steps

  Step 1: estimate the missing value in the simulation data set by using the missing value estimation method [23] and construct the complete dataset.
  Step 2: calculate the time-delay relative change trend coefficient matrix, the time-delay correlation coefficient matrix, and the time-delay mutual information matrix of all gene pairs in the complete dataset.
  Step 3: obtain the similarity evaluation matrix of gene pair. This similarity evaluation matrix is a multidimensional space matrix. For simulation simplicity, the matrix is processed accordingly to be converted to the two-dimensional space matrix. Make *I*=(*i*_*m*′*f*_′)_(*A* × *c*_*N*_^2^)×3_, wherein the row sequence of the row vector *i*_*m*′_′ is as follows: no delay between the gene 1 and the gene 1, delay 1 time unit between the gene 1 and the gene 1, and delay *A* time unit between the gene *N* and the gene *N*.
  Step 4: add the label value to a small number of gene pairs, calculate the fuzzy label values of unknown gene pairs on the basis of fuzzy label propagation algorithm, and obtain the regulation relationship and the time delay between the genes.

### 4.3. Time Complexity Analysis of Algorithm

There are two main bottlenecks in the calculation of this algorithm. The first is to use mutual information to find the time delay between gene pairs, and the second is to use fuzzy label transfer algorithm to classify datasets. It is assumed that the number of genes is *N*, the length of gene time series is *T*, the maximum time delay is *m*, and the number of iterations of fuzzy label transfer algorithm is *M*. When we use equation (6) to find the mutual information of a target gene and its regulator under a certain time delay, we need to traverse the gene expression level matrix once, and the algorithm complexity is *O*(*N∗T*). So, the time complexity of the algorithm is *O*(*N*^2^*Tm*). The time complexity of initialization is *O*(*N*^2^). The time complexity of fuzzy label transfer algorithm using semisupervised learning is *O*(*M*). The time complexity of calculating score function is *O*(*NT*). Therefore, the total time complexity is *O*(*N*^2^*Tm*+*MNT*).

## 5. Results and Discussion

### 5.1. Simulation Dataset

The simulation dataset is selected from the yeast cell gene chip data [24, 25] provided by Spellman et al. in Stanford University, from which 6 genes are extracted to form a small gene regulation network. The data are as shown in Table 1.

Extract the regulation relationship among 6 genes based on the research of Hou et al. [26]. The regulation network structure is shown in Figure 1.

## 6. Results

In simulation, firstly we need to select part of samples to add the labels. In this paper, the sample label value is set to −1 when the delay between the genes Clb6 and Cln1 is 0, the sample label value is set to 1 when the delay between the genes Clb2 and Cln2 is 0, and the maximum time delay *A* is set to 2. The simulation results are shown in Table 2.

It can be seen from Figure 1 that there are 10 pairs of genes having the regulation relationship. Table 2 shows that the method of this paper can correctly identify 8 pairs of genes having the regulation relationship, accounting for 80% of the total gene pairs having the regulation relationship, and the accuracy is relatively perfect. In 8 pairs of genes correctly identified, there are two pairs of genes having time delay, namely, Swi5 and Cln2 and Cln2 and Clb1, and the time delay is 1 unit. The change relationship of expression values for 8 pairs of genes correctly identified is shown in Figure 2. Horizontal coordinates represent gene expression level and vertical coordinates represent time point of gene expression.

It can be seen from Figure 2 that the change relationships of the gene expression data in Figures 2(a) and 2(c)–2(e) are basically consistent and the change relationships of the gene expression data in Figures 2(b) and 2(f)–2(h) are basically contrary, and Figure 2(g) shows the change relationship between the gene Cln2 and the gene Clb1 after the gene Cln2 is delayed by 1 unit of time. On the left side, the time points corresponding to the peaks and troughs of Cln2 expression value and Clb1 expression value are basically the same, and the change trends are contrary; on the right side, the expression value changes of two genes are disordered to some extent, but except for the last three time points, the expression value changes of other time points substantially conform to the change contrary trends.  Figure 2(h) shows the expression value change relationship between the gene Cln2 and the gene Swi5 after the gene Cln2 is delayed by 1 unit of time. It can be seen from the figure that the change trends of two gene expression values are contrary, wherein the first peak of the expression value for the gene Swi5 was obtained at the seventh time point and the first trough of the expression value for the gene Swi5 was obtained at the twelfth time point; the first peak of the expression value for the gene Cln2 was obtained at the seventh time point, and the first trough of the expression value for the gene Cln2 was obtained at the eleventh time point; the time points of peaks and troughs for the two genes are basically the same. Therefore, based on the premise and assumption, the result that the time delay between Swi5 and Cln2 and between Cln2 and Clb1 is 1 time interval in the regulation is reasonable.

## 7. Discussion

In order to have objective and scientific comparison results, hypothesis testing is used on the experimental results. Let the variables *X*_1_, *X*_2_, *X*_3_, *X*_4_ denote the classification error rate of algorithms proposed in this paper, reference [17], reference [20], and reference [27], respectively. Since the value of *X*_1_, *X*_2_, *X*_3_, *X*_4_ is subject to many random factors, we assume that they submit to normal distribution, *X*_*i*_ ~ *N*(*μ*_*i*_, *σ*_*i*_^2^), *i*=1,2,3,4. Now, we compare the random variable mean of these algorithms, *μ*_*i*_ (*i*=1,2,3,4). The smaller *μ*_*i*_ is, the lower the expected classification error rate is and the higher the efficiency is. Because the sample variance is the unbiased estimation of the overall variance, the sample variance value is used as an estimate of the generality variance. In this experiment, the significance level *α* is set as 0.01.

Table 3 shows the comparison process on *μ*_*i*_ and other parameters. We can see from Table 1 that the expectations of classification error rate in this paper are far below than other algorithms.

Next, we use some evaluation indexes to evaluate the algorithm. TP, TN, FP, and FN are abbreviations of true positive, false positive, true negative, and false negative, respectively. Perform the following operations on all target genes and regulatory genes. If the regulatory relationship between the target gene and regulatory gene is inferred by this algorithm and the previous literature has proved the regulatory relationship, then the value of TP is increased by 1. If the regulatory relationship between the target gene and regulatory gene is inferred by this algorithm, but the previous literature has not proved the regulatory relationship, then FP is increased by 1. If the algorithm in this paper does not infer the regulatory relationship between the target gene and the regulatory gene and no previous literature has proved that there is a regulatory relationship between the target gene and the regulatory gene, then the value of TN is increased by 1. And if the algorithm in this paper does not infer that there is a regulatory relationship between the target gene and the regulatory gene, but the previous literature has proved that the regulatory relationship exists, then add 1 to the value of FN. Each algorithm evaluation standard is evaluated by some combination of TP, FP, TN, and FN. The most common algorithms for predicting gene regulatory networks are sensitivity (Sn), specificity (Sp), and accuracy (Acc). Sn = TP/(TP + FN), Sp = TN/(TN + FP), and Acc = (TP + TN)/(TP + FP + TN + FN). The comparison results are shown in Table 4.

Table 4 compares the inference results of the four methods for gene regulatory network. The sensitivity of reference [17] method is only 37.5%, that of reference [20] method is 36.4%, that of reference [27] method is 24.2%, and that of the proposed method is 43.8%. It can be seen that in the network construction of this gene, the method proposed in this paper is better for identifying the right edge; it also shows that the addition of transcription factor linkage site data reduces the information loss in data processing. The data in accuracy are also optimal, which shows that the accuracy of network construction in this paper has been improved.

Therefore, each gene has a complex regulatory relationship in different cell cycles. The direction of regulation can be determined by using the method of multiple time delay, which is in line with the mechanism of biological time sequence activity. The introduction of transcription factor linked site data can reduce the network complexity and construct the regulatory network more effectively.

To sum up, the multi-time-delay gene regulation network method based on the fuzzy label propagation is feasible.

## 8. Conclusions

In consideration of the time delay existing in the interaction of genes, this paper constructs the multi-time-delay gene regulation network, uses the relative change trend coefficient, the correlation coefficient, and the mutual information as the evaluation indexes of the gene pair to construct the similarity matrix of the gene pairs, and then analyses the regulation relationship and the time delay among the genes by using the fuzzy label propagation algorithm. Due to the high complexity of algorithm in this paper, the method proposed in this paper is unsuitable for the construction of large network, and the error recognition ratio will be increased when the maximum time delay is set to high value. However, the method proposed in this paper is feasible. Therefore, how to effectively modularize the large network, divide the large network into many small networks, and integrate the small networks into the large network in the analysis will be an improvement direction of the method in this paper.

## Figures and Tables

**Figure 1:** The structure of regulatory network formed by the 6 genes.

**Figure 2:** The changing relationship of the eight gene pairs. (a) The changing relationship of Cln1 and ln2. (b) The changing relationship of Cln2 and Clb2. (c) The changing relationship of Clb1 and Swi5. (d) The changing relationship of Clb2 and Swi5. (e) The changing relationship of Clb1 and sClb2. (f) The changing relationship of Cln1 and Clb2. (g) The change relationship between Cln2 and Clb1 after Cln2 is delayed by 1 unit of time. (h) The change relationship between Cln2 and Swi5 after Cln2 is delayed by 1 unit of time.

**Table 1:** The information of selected genes.

Gene	Dataset	Gene	Dataset	Gene	Dataset
Cln1	YMR199W	Clb2	YPR119W	Clb1	YGR108W
Cln2	YPL256C	Clb6	YGR109C	Swi5	YDR146C

**Table 2:** The correctly identified gene pairs and the time delay.

Gene pairs	Cln1-Cln2	Swi5-Cln2	Swi5-Clb2	Cln2-Clb2	Cln1-Clb2	Cln2-Clb1	Swi5-Clb1	Clb2-Clb1
Time delay	0	1	0	0	0	1	0	0

**Table 3:** Hypothesis testing for experimental results.

Hypothesis	$\begin{array}{c} H_{0}\;:\;\mu_{1}\geq \mu_{2}\\ H_{1}\;:\;\mu_{1}<\mu_{2} \end{array}$	$\begin{array}{c} H_{0}\;:\;\mu_{1}\geq \mu_{3}\\ H_{1}\;:\;\mu_{1}<\mu_{3} \end{array}$	$\begin{array}{c} H_{0}\;:\;\mu_{1}\geq \mu_{4}\\ H_{1}\;:\;\mu_{1}<\mu_{4} \end{array}$
Statistics	$U_{1}=\left({\bar{X}}_{1}-{\bar{X}}_{2}\right)/\left(\sqrt{\left(\sigma_{1}^{2}/n_{1}\right)+\left(\sigma_{2}^{2}/n_{2}\right)}\right)$	$U_{2}=\left({\bar{X}}_{1}-{\bar{X}}_{3}\right)/\left(\sqrt{\left(\sigma_{1}^{2}/n_{1}\right)+\left(\sigma_{3}^{2}/n_{3}\right)}\right)$	$U_{3}=\left({\bar{X}}_{1}-{\bar{X}}_{4}\right)/\sqrt{\left(\sigma_{1}^{2}/n_{1}\right)+\left(\sigma_{4}^{2}/n_{4}\right)}$

Rejection region	*U*_1_ ≤ −*Z*_*α*_=−2.325	*U*_2_ ≤ −*Z*_*α*_=−2.325	*U*_3_ ≤ −*Z*_*α*_=−2.325

Value of the statistic	*U*_1_=−36.24	*U*_2_=−58.32	*U*_3_=−76.65

Conclusion	*H*_1_ : *μ*_1_ < *μ*_2_	*H*_1_ : *μ*_1_ < *μ*_3_	*H*_1_ : *μ*_1_ < *μ*_4_

**Table 4:** Comparison between the methods in this paper and other methods.

Algorithm	TP	TN	FP	FN	Sn (%)	Sp (%)	Acc (%)
Reference [17]	12	185	27	20	37.5	87.3	80.7
Reference [20]	12	183	28	21	36.4	86.7	79.9
Reference [27]	8	180	31	25	24.2	85.3	77.0
This paper	14	187	25	18	43.8	88.2	82.4

## Data Availability

The yeast cell gene chip data used to support the findings of this study have been deposited by Spellman et al. in Stanford University.
